This article has been retracted.

# Overexpression of long intergenic noncoding RNA LINC00312 inhibits the invasion and migration of thyroid cancer cells by down-regulating microRNA-197-3p

**DOI:** 10.1042/BSR20170109

**Published:** 2017-07-20

**Authors:** Kai Liu, Wen Huang, Dan-Qing Yan, Qing Luo, Xiang Min

**Affiliations:** 1 Department of Otorhinolaryngology and Head and Neck Surgery, The First Affiliated Hospital of Nanchang University, Nanchang 330006, P.R. China; 2 Department of Blood Transfusion, The First Affiliated Hospital of Nanchang University, Nanchang 330006, P.R. China

**Keywords:** Cell migration, invasion and migration, Long intergenic noncoding RNA LINC00312, MicroRNA-197-3p, proliferation, Thyroid cancer

## Abstract

The study evaluated the ability of long intergenic noncoding RNA LINC00312 (LINC00312) to influence the proliferation, invasion, and migration of thyroid cancer (TC) cells by regulating miRNA-197-3p. TC tissues and adjacent normal tissues were collected from 211 TC patients. K1 (papillary TC), SW579 (squamous TC), and 8505C (anaplastic TC) cell lines were assigned into a blank, negative control (NC), LINC00312 overexpression, *miR-197-3p* inhibitors, and LINC00312 overexpression + *miR-197-3p* mimics group. The expression of LINC00312, *miR-197-3p*, and p120 were measured using quantitative real-time PCR (qRT-PCR) and Western blotting. Cell proliferation was assessed via CCK8 assay, cell invasion through the scratch test, and cell migration via Transwell assay. In comparison with adjacent normal tissues, the expression of LINC00312 is down-regulated and the expression of *miR-197-3p* is up-regulated in TC tissues. The dual luciferase reporter gene assay confirmed that P120 is a target of *miR-197-3p*. The expression of LINC00312 and p120 was higher in the LINC00312 overexpression group than in the blank and NV groups. However, the expression of *miR-197-3p* was lower in the LINC00312 overexpression group than in the blank and NC groups. The *miR-197-3p* inhibitors group had a higher expression of *miR-197-3p*, but a lower expression of p120 than the blank and NC groups. The LINC00312 overexpression and *miR-197-3p* inhibitor groups had reduced cell proliferation, invasion and migration than the blank and NC groups. These results indicate that a LINC00312 overexpression inhibits the proliferation, invasion, and migration of TC cells and that this can be achieved by down-regulating *miR-197-3p*.

## Introduction

Thyroid cancer (TC) accounts for only 1% of all the malignancies and is a common endocrine malignancy, which is derived from follicular thyroid or parafollicular C cells [1]. In China in 2000, the incremental incidence and mortality rates of TC in patients below 74 years were 0.32 and 0.03%, respectively [2]. The overall 10-year survival rate of differentiated TC is above 80%, 5–20% of patients develop local or regional recurrences and 10–15% develop distant metastases [3]. Conventional surgery such as adjuvant ablation by radioiodine treatment has been the main therapy for TC. In most cases, however, it is often incurable [1]. Identifying genetic factors can facilitate the treatment and prevention of TC, but the ideal genetic marker for TC detection has not yet been identified [4]. Recently, researchers have attempted to explore long noncoding RNAs (lncRNAs) as a possible regulator in tumorigenesis and tumor development. To date, only a few lncRNAs such as lncRNA PTCSC3, lncRNA NAMA, and lncRNA BANCR have been proven to be involved in TC development and progression [5–7].

LncRNAs have little to no protein coding ability, transcripts which exhibit cell-type specific expression, localization of subcellular compartments, or correlation with human diseases. Many lncRNAs are processed to yield small RNAs [8]. Long intergenic noncoding RNA LINC00312 (LINC00312), also known as NAG7, is a long intergenic noncoding RNA located on 3p25.3 and has been demonstrated to be a novel putative tumor suppressor gene [9]. Subsequently, it has been reported that LINC00312 may act as a potential biomarker for metastasis, progression, and prognosis in nasopharyngeal carcinoma [10]. In addition, miRNAs are small noncoding RNAs which can affect tumorigenesis through different mechanisms [11]. *miR-197-3p* belongs to *miR-197* family and has been demonstrated to have a low expression in primary biliary cirrhosis [12]. In basal cell carcinoma, *miR-197-3p* is usually overexpressed, and can inhibit keratinocyte proliferation and migration [13]. LINC00312 has been reported to have a negative correlation with *miR-197-3p* in bladder cancer. It has also been reported that LINC00312 can inhibit the invasion and metastasis of bladder cancer cell by down-regulating *miR-197-3p* [14]. LncRNAs and miRNAs have been found to be significantly associated with TC. For example, lncRNA H19 regulates YES1 expression by binding *miR-17-5p* and *miR-146a* polymorphism predisposing patients to TC [15,16]. However, the effects of LINC00312 and *miR-197-3p* have not been proven on TC. Therefore, this research was conducted to investigate the involvement of LINC00312 and *miR-197-3p* in TC and demonstrate their effect on the proliferation, invasion, and migration ability of TC cells.

## Materials and methods

### Ethical statement

The study was approved by the ethical committee of the First Affiliated Hospital of Nanchang University. All research tissues were obtained from patients who had signed informed consent forms.

### Study subjects

The study included 211 TC tissues and 70 adjacent normal tissues (2 cm away from the tumor site) obtained from 211 TC patients (99 females and 112 females) who were diagnosed with TC. All patients received primary surgical resection at the First Affiliated Hospital of Nanchang University between October 2013 and August 2015. All the samples were confirmed via pathological examination, all patients had not received any previous treatment and had no severe systemic diseases such as malignant tumors or severe systemic infections. The average age of patients was 46.43 ± 14.27 years (ranging from 20 to 75 years). According to the tumor node metastasis (TNM) staging standards [17] published by the Union for International Cancer Control (UICC), there were 190 patients in phase I/II and 21 patients in phase III/IV [17]. Sixty-nine patients had lymph node metastasis and 142 patients did not show lymph node metastasis. Seventy-two patients had tumor diameter ≥1.0 cm and 139 patients had tumor diameter <1.0 cm. One hundred and eight patients had papillary TC, 54 patients had follicular TC, 36 patients had squamous TC, and 13 patients had anaplastic TC. The samples were preserved at –70°C for further use.

### Cell culture

K1 (papillary TC), SW579 (squamous TC), and 8505C (anaplastic TC) cell lines (Chinese Academy of Sciences, Shanghai, China) were used in our study. Cells were cultured in Dulbecco’s modified Eagle’s medium (DMEM) (Promega, Madison, WI, U.S.A.) containing 15% FBS (HyClone, Logan, Utah, U.S.A.) and 1% streptomycin at 37°C with 95% relative humidity and 5% CO_2_. Cells with 80% adherence were used for subculturing. Cells were then rinsed twice with PBS and digested with trypsin (Gibco Company, Grand Island, NY, U.S.A.). The trypsin was removed when the intercellular space was enlarged. Cells were routinely passaged without suspension cells in the above-mentioned culture medium.

### Luciferase reporter gene assay

The potential target gene and fragment sequences containing *miR-197-3p* reaction sites were analyzed using microRNA.org. The DNA was extracted in strict accordance with the instructions of the TIANamp Genomic DNA Kit (Tiangen Biotech, Beijing, China). The p120 3′-UTR wild-type (WT) sequence named p120-3′-UTR-WT was 5′-CACTTTTATTTTTTGGTGGTGAAT-3′ and the mutant sequence of p120 3′-UTR missing the binding site with *miR-197-3p* named p120-3′-UTR-Mut was 5′-CACTTTTATTTTTTGACAAGTCCT-3′. The luciferase reporter gene vector was constructed and TC cells were transfected. Luciferase reporter gene assay kits (Promega, Madison, WI, U.S.A.) were used to detect the luciferase activity of samples. At 48 h after transfection, the culture medium was removed and the samples were washed twice with 0.1 M PBS (8 g NaCl, 0.2 g KCl, 3.58 g Na_2_HPO_4_.12H_2_O, and 0.24 g KH_2_PO_4_ mixed and dissolved with double distilled water to 100 ml, pH 7.4). Passive lysis buffer (100 μl) was added into each well. Samples were slightly oscillated at room temperature for 15 min and then the cell lysis buffer was collected. Two seconds of prereading was conducted before 10 s of reading. The sample volume of Luciferase Assay Reagent II (LARII) and Stop & Glo® Reagent was 100 μl. The luminotron or luminous plate (20 μl per sample) which had been added with LARII and Stop & Glo® Reagent was placed into the biological luminous detector (type Modulus™, Turner BioSystems, Inc., Sunnyvale, CA, U.S.A.).

### Cell transfection and grouping

The primer sequences of the negative control (NC) plasmid, *miR-197-3p* inhibitors plasmid, and LINC00312 overexpression + *miR-197-3p* mimics plasmid were constructed by Sangon Biotech, Shanghai, China (Table 1) based on the *miR-197-3p* sequence issued by National Center for Biotechnology Information. After trypsin digestion, the second-generation cells were seeded into a 24-well plate and the culture medium was abandoned after the cells displayed monolayer growth. The cells were divided into a blank (no transfection), NC (cells transfected with NC plasmids), LINC00312 overexpression (cells transfected with LINC00312 overexpression plasmids), *miR-197-3p* inhibitors (cells transfected with *miR-197-3p* inhibitor plasmids), and LINC00312 overexpression + *miR-197-3p* mimics group (cells transfected with LINC00312 overexpression + *miR-197-3p* mimic plasmids).

**Table 1:** Primer sequences for NCs, *miR-197-3p* mimics, and *miR-197-3p* inhibitors

Target fragments	Sequence
NCs	5′-CAGUACUUUUGUGUAGUACAA-3′
*miR-197-3p* mimics	5′-UUCACCACCUUCUCCACCCAGC-3′
*miR-197-3p* inhibitors	5′-GCUGGGUGGAGAAGGUGGUGAA-3′

### Quantitative real-time PCR

Total RNA was extracted from cancer tissues and adjacent normal tissues using the TRIzol standard method (Invitrogen, Carlsbad, CA, U.S.A.). Isolated RNA was dissolved in 0.1% diethylpyrocarbonate water (Fermentas, Glen Burnie, MD, U.S.A.) and then optical density (OD) at 260/280 nm and RNA quality were determined. Primer sequences design is shown in Table 2. Reverse transcription and PCR were also conducted in accordance with the manufacturer’s instructions. Reverse transcription was carried out three times as follows: 10 min at 74°C, 2 min of ice bathing, 60 min at 42°C, and 10 min at 70°C. PCR was performed three times in the following sequence: predenaturation at 95°C for 1 min, followed by 40 cycles at 95°C for 15 s, 60°C for 30 s, and 72°C for 30 s. The relative expression of target genes were calculated using the 2^−ΔΔ*C*^_t_ method with U6 as the internal reference for *miR-197-3p* and β-actin for other target genes. Each experiment was repeated three times.

**Table 2:** Primer sequences of LINC00312, *miR-197-3p*, p120, U6, and β-actin for quantitative real-time PCR

Gene	Sequence
*LINC00312*	F: 5′-AAGCGAACCAAGCCAATA-3′
	R: 5′-CAAATCCCTGAAACTCTG-3′
*miR-197-3p*	F: 5′-AGTTGTTCACCACCTTCTCCAC-3′
	R: 5′-TATCGTTGTACTCCAGTCCAAGTC-3′
*p120*	F: 5′-GGACACCCTCTGACCCTCG-3′
	R: 5′-GCTTGCTAAACTTCCTCGCTC-3′
*U6*	F: 5′-GTGCTCGCTTCGGCAGCACATATAC-3′
	R: 5′-AAAAATATGGAACGCTCACGAATTTG-3′
*β-actin*	F: 5′-CAGCAAGCAGGAGTATGACG-3′
	R: 5′-GAAAGGGTGTAACGCAACTAA-3′

Abbreviations: F, forward; R, reverse.

### Western blotting

Cell samples were washed with precooled 0.1 M PBS and then lysed with cell lysis solution (RIPA). Ice bathing was conducted for 30 min, followed by centrifugation at 12000 rpm at 4°C for 10 min. The supernatant was collected and preserved at –20°C for further use. BSA (2 μg/μl) was diluted with 0.1 M PBS to the following concentrations: 20, 15, 10, 5, 2.5, and 0 μg/ml. Protein concentration was detected using BCA (Thermo Fisher Scientific Inc., MA, U.S.A.) according to the instructions and sample numbers. The protein was electrophoresed in a 4°C chromatography cabinet with 80 V of compressive gel and 120 V of separation gel. The electrophoresed proteins were transferred on to a PVDF membrane, blocked in TBST (25 mM Tris, 140 mM NaCl, and 0.1% Tween 20, pH 7.5) containing 5% skimmed milk and incubated for 2 h. The proteins were combined with the primary antibody of p120 (1:500; article number ab10297; Abcam Inc., Cambridge, MA, U.S.A.) and β-actin (1:10000; article number ab8226; Abcam Inc., Cambridge, MA, U.S.A.) and incubated at 4°C overnight. After being washed (3 × 10 min) with TBST, the secondary antibody was added and incubated at room temperature for 1 h. Subsequently, the cells were rewashed with TBST (3 × 10 min) and chemiluminescence was conducted. The results were analyzed according to the developed and fixed X-ray films.

### CCK8 assay

Cells in the logarithmic phase of each group were digested with trypsin to regulate cell concentration. Cells were seeded into six-well plates (1 × 10^5^ cells/well), cultured in an incubator (Heal Force HF90, Healforce Biomedical Technology Holding Group, Hongkong, China) for 24 h and then transfected. Subsequently, the cells were digested with trypsin and the cell culture medium was collected and placed into centrifuge tubes. Once the cell concentration reached 3 × 10^5^/ml, cells were seeded in four 96-well plates (3000 cells/well). Four groups were set in each plate, and four replicates were set in each group. The samples were incubated in culture plates with 5% CO_2_ at 37°C. The culture plates were placed in an incubator and were taken out after 24, 48, 72, and 96 h. CCK8 solution (10 μl, Sigma, SF, U.S.A.) was added into each well (no bubbles were observed when the mixture was combined). The culture plates were placed in an incubator at 37°C with 5% CO_2_ for 2 h. The absorption value was measured at 450 nm using a microplate reader (Bio-Rad, Cal, U.S.A.). The experiment was repeated three times.

### Transwell assay

The wells in the upper chamber were coated with 30 μl of Matrigel (dissolved overnight, diluted with FBS-free DMEM in triplicate volume and added at a 15-min interval). Each well in the upper chamber was inoculated with 2 × 10^4^ cells. DMEM (0.5 ml) containing 10% FBS was added into each well of the lower chamber. After 24 h of incubation, the cells were fixed with paraformaldehyde and stained with 0.1% Crystal Violet for 0.5 h to remove any uninfected cells from the upper chamber. Next, cells were washed with 0.1 M PBS, counted and photographed in randomly selected fields with a light microscope. The experiment was repeated three times. The mean value of cells which penetrated through the Matrigel was analyzed to determine the cells’ migration ability.

### Scratch test

Cells were seed into a 12-well plate with 1.0 × 10^4^ cells in each well. Three parallel lines were made on the back of each well. After the well was completely covered with cells, the confluent monolayer of each well was scratched with a pipette tip. Cells were then washed with 0.1 M PBS and cultured in a medium. Cells were photographed under a light microscope after 0 and 48 h. The cell position at 0 h was used as the reference point. The relative scratch width of cancer cells was recorded and analyzed to detect the cancer cells invasion ability. The experiment was repeated at least three times.

### Tumor xenograft in nude mice

TC cells in the logarithmic phase were digested with trypsin to obtain cell suspension. The number of cells was observed with an optical microscope and then cells were collected and preserved at −20°C for further use. Fifty 6–8 week old healthy nude mice (Hunan SJA Laboratory Animal Co. Ltd, Changsha, China) were randomly divided into three groups with five mice in each group. The mice were injected with the transfected cell suspension (1 × 10^5^ cells) subcutaneously and then fed conventionally. After the tumor formation, its size (length, width, and height) was roughly calculated every 2 days. After 3 weeks, the mice were killed via cervical dislocation and photos were taken.

### Statistical analysis

The SPSS 21.0 software (SPSS Inc., Chicago, IL, U.S.A.) was utilized for data analysis. Measurement data are expressed as mean ± S.D. and the comparison between the two groups was measured using the independent *t* test. One-way ANOVA was used to compare multiple groups and LSD-t was adopted for pairwise comparisons. A *P*-value less than 0.05 is considered statistically significant.

## Results

### Expression levels of LINC00312 and *miR-197-3p* in TC and adjacent normal tissues

The expression levels of LINC00312 and *miR-197-3p* in TC tissues and adjacent normal tissues were detected via quantitative real-time PCR (qRT-PCR). Figure 1A demonstrates that the expression level of LINC00312 in TC tissues (1.02 ± 0.33) is significantly lower than that of the adjacent normal tissues (3.89 ± 0.58) (*P*<0.05). Figure 1B displays that *miR-197-3p* is significantly higher in TC tissues (2.94 ± 0.65) (*P*<0.05) than in adjacent normal tissues (1.41 ± 0.36).

**Figure 1:** Comparison of expression levels of LINC00312 (**A**) and *miR-197-3p* (**B**) in the TC tissues (*n*=211) and adjacent normal tissues (*n*=70) by qRT-PCR (mean ± S.D.). *, *P*<0.05 compared with the adjacent normal tissues.

### Correlation between the expression level of LINC00312 and *miR-197-3p* and the clinicopathological characteristics of TC patients

Table 3 highlights that LINC00312 expression is significantly lower in patients with anaplastic TC, lymph node metastasis, tumors in stage III/IV, or have tumor diameter ≥1.0 cm (all *P*<0.05). The expression level of *miR-197-3p* is significantly higher in patients with anaplastic TC, lymph node metastasis, tumors in stage III/IV, or have tumor diameters ≥1.0 cm (all *P*<0.05). No association was found between the relative expression of LINC00312 or *miR-197-3p* with the age or gender of patients (all *P*>0.05).

**Table 3:** Correlation between the expression levels of LINC00312 and *miR-197-3p* with clinicopathological characteristics of TC patients (*n*=211, mean ± S.D.)

Clinicopathological characteristics	Cases	LINC00312	*P*	*miR-197-3p*	*P*
Age (years)					
<50	108	1.06 ± 0.36	0.082	2.95 ± 0.53	0.912
≥50	103	0.98 ± 0.30		2.94 ± 0.76	
Gender					
Male	99	1.04 ± 0.39	0.513	3.02 ± 0.62	0.092
Female	112	1.01 ± 0.27		2.87 ± 0.66	
TNM					
I/II	190	1.07 ± 0.29	<0.001	2.85 ± 0.54	<0.001
III/IV	21	0.62 ± 0.39		3.80 ± 0.87	
Lymph node metastasis					
No	142	1.08 ± 0.32	<0.001	2.81 ± 0.61	<0.001
Yes	69	0.90 ± 0.33		3.21 ± 0.65	
Tissue-type					
Papillary TC	108	1.16 ± 0.26	Ref.	2.70 ± 0.64	Ref.
Follicular TC	54	1.02 ± 0.31	0.003	2.95 ± 0.27	0.006
Squamous TC	36	0.77 ± 0.24	<0.001	3.32 ± 0.55	<0.001
Anaplastic TC	13	0.56 ± 0.36	<0.001	3.88 ± 0.82	<0.001
Tumor diameter (cm)					
<1.0	139	1.09 ± 0.32	<0.001	2.79 ± 0.60	<0.001
≥1.0	72	0.90 ± 0.33		3.24 ± 0.64	

### P120 was confirmed to be a target of *miR-197-3p*

The targetted site at which p120 combined with *miR-197-3p* was predicted using the online software TargetScan. Figure 2A shows the binding sequences of 3′-UTR (where the p120 mRNA combines with *miR-197-3p*). TC cells were transfected with *miR-197-3p* mimics and WT-*miR-197-3p*/p120 or Mut-*miR-197-3p*/p120 recombinant plasmids. The results indicate that *miR-197-3p* mimics have no significant effect on the luciferase activity of Mut-*miR-197-3p*/p120 plasmids (0.93 ± 0.03) (*P*>0.05). However, they decreased the luciferase activity of the WT-*miR-197-3p*/p120 plasmid (0.35 ± 0.09) by 65% (*P*<0.05) (Figure 2B).

**Figure 2:** Target relations between *miR-197-3p* and p120 gene (mean ± S.D.) (**A**) *MiR-197-3p* combined with p120 3′-UTR; (**B**) luciferase activity of p120 WT and p120 Mut; *, *P*<0.05, compared with the control; four wells of cells in each group were repeated and the experiment was repeated for three times.

### Expression levels of LINC00312, *miR-197-3p*, p120 in K1, SW579, and 8505C cells after transfection

The expression levels of LINC00312, *miR-197-3p*, p120 in the K1, SW579, and 8505C cell lines were detected and are displayed in Figure 3. In the 8505C cell line, the expression level of LINC00312 was 0.78 ± 0.13, the mRNA level of p120 was 0.73 ± 0.17 and the protein level of p120 was 1.09 ± 0.12. In the K1 cell line, the expression level of LINC00312 was 1.62 ± 0.18, the mRNA level of p120 was 1.27 ± 0.12, and the protein level of p120 was 2.44 ± 0.36. In the SW579 cell line, the expression level of LINC00312 was 1.21 ± 0.12, the mRNA level of p120 was 1.01 ± 0.11, and the protein level of p120 was 2.01 ± 0.21 (all *P*<0.05). The expression level of *miR-197-3p* in the 8505C, K1, and SW579 cell lines was 1.93 ± 0.11, 0.84 ± 0.09, and 1.21 ± 0.10, respectively (all *P*<0.05). Results of the three cell lines in the other groups were very similar. For example, in the K1 cell line, the expression levels of LINC00312, *miR-197-3p*, and the mRNA level of p120 in the blank group was 1.08 ± 0.12, 1.74 ± 0.19, and 0.86 ± 0.09, respectively. In the NC group, the expression levels of LINC00312, *miR-197-3p*, and the mRNA level of p120 was 1.02 ± 0.08, 1.78 ± 0.12, and 0.84 ± 0.08, respectively. There was no significant difference between the two groups (all *P*>0.05). The expression level of LINC00312 in the LINC00312 overexpression group was 1.62 ± 0.18. In the INC00312 + *miR-197-3p* mimics group, it was 1.64 ± 0.11. Both these results were higher than the blank group (1.08 ± 0.12) (all *P*<0.05). There were no significant differences in the expression level of LINC00312 between blank and *miR-197-3p* inhibitor groups. The expression level of *miR-197-3p* in the LINC00312 overexpression (0.84 ± 0.09) and *miR-197-3p* inhibitors group (0.88 ± 0.08) was significantly lower (all *P*<0.05) than the blank (1.74 ± 0.19) and NC group (1.78 ± 0.12). There was no significant difference in the expression of *miR-197-3p* between the blank (1.74 ± 0.19) and LINC00312 overexpression + *miR-197-3p* mimics groups (1.71 ± 0.11). In comparison with the blank (0.86 ± 0.09 and 1.93 ± 0.29) and NC groups (0.84 ± 0.09 and 1.76 ± 0.28), the expression level of p120 was higher in the LINC00312 overexpression (1.27 ± 0.12 and 2.44 ± 0.36) and *miR-197-3p* inhibitors groups (1.35 ± 0.20 and 2.48 ± 0.38) (all *P*<0.05). There was no significant difference in the expression of p120 in the blank and LINC00312 overexpression + *miR-197-3p* mimic groups (0.79 ± 0.08 and 1.85 ± 0.31). The expression level of K1 cell line in the LINC00312 group was much higher than that of the LINC00312 + *miR-197-3p* mimics group. The results of the other two cell lines were in-line with the results of the K1 cell line.

**Figure 3:** The expression levels of LINC00312, *miR-197-3p*, and p120 amongst different TC cells detected by qRT-PCR and Western blotting (mean ± S.D.) (**A**)The expression levels of LINC00312 and *miR-197-3p*, and the mRNA level of p120; (**B**) protein band patterns of p120 amongst different TC cells; the first row from top to bottom, the gray value of p120 protein band in K1 cells; the second row, the gray value of β-actin band in K1 cells; the third row, the gray value of p120 protein band in SW579 cells; the fourth row, the gray value of β-actin band in SW579 cells; the fifth row, the gray value of p120 protein band in 8505C cells; the sixth row, the gray value of β-actin band in 8505C cells; (**C**) the protein level of p120 by Western blotting; *, *P*<0.05, compared with the blank group; ^#^, *P*<0.05, compared with the NC group; ^&^, *P*<0.05, compared with the LINC00312 overexpression + *miR-197-3p* mimics group; four wells of cells in each group were repeated, and the experiment was repeated for three times.

### LINC00312 inhibits K1, SW579, and 8505C cell proliferation by down-regulating *miR-197-3p*

The proliferation of K1, SW579, and 8505C cells was measured via CCK8 assay (Figure 4). The OD value of the TC cell lines at 48, 72, and 96 h after transfection demonstrate that 8505C cells have the strongest proliferation ability (0.38 ± 0.02, 0.60 ± 0.03, and 0.70 ± 0.03). The proliferation ability of K1 cells was the weakest (0.13 ± 0.02, 0.25 ± 0.03, and 0.32 ± 0.03) and the proliferation ability of SW579 cells was in between (0.23 ± 0.03, 0.47 ± 0.05, and 0.65 ± 0.04) (all *P*<0.05). The other groups also displayed similar results. For example, in the K1 cell line, there were no significant differences between the blank (0.21 ± 0.02, 0.39 ± 0.04, and 0.47 ± 0.04), NC (0.22 ± 0.04, 0.42 ± 0.03, and 0.49 ± 0.03) and LINC00312 + *miR-197-3p* mimics groups, 48, 72, and 96 h after transfection (*P*>0.05). The proliferation ability was significantly lower in the LINC00312 overexpression (0.13 ± 0.02, 0.25 ± 0.03, and 0.32 ± 0.03) and *miR-197-3p* inhibitors (0.12 ± 0.02, 0.21 ± 0.03, and 0.27 ± 0.04) groups 48, 72, and 96 h after transfection than the blank (0.21 ± 0.02, 0.39 ± 0.04, and 0.47 ± 0.04) and NC (0.22 ± 0.04, 0.42 ± 0.03, and 0.49 ± 0.03) groups. The proliferation ability of the LINC00312 overexpression group (0.13 ± 0.02, 0.25 ± 0.03, and 0.32 ± 0.03) was significantly weaker than that of the LINC00312 + *miR-197-3p* mimics group (0.23 ± 0.04, 0.38 ± 0.04, and 0.48 ± 0.04) (all *P*<0.05). The results of the other two cell lines were in-line with the K1 cell line. The results indicated that LINC00312 inhibits K1, SW579, and 8505C cell proliferation by down-regulating *miR-197-3p*.

**Figure 4:** Proliferation abilities of K1, SW579, and 8505C cells amongst five groups (mean ± S.D.) *, *P*<0.05, compared with the blank group; ^#^, *P*<0.05, compared with the NC group; ^&^, *P*<0.05, compared with the LINC00312 overexpression + *miR-197-3p* mimics group; four wells of cells in each group were repeated, and the experiment was repeated for three times.

### LINC00312 suppresses K1, SW579, and 8505C cell invasion by down-regulating *miR-197-3p*

The invasion ability of cells was detected 24 h after transfection. As shown in Figure 5, the number of invasive cells in the blank, NC, LINC00312 overexpression, *miR-197-3p* inhibitors, and LINC00312 overexpression + *miR-197-3p* mimics groups in the K1 cell line (the same below) was 114.67 ± 15.13, 99.49 ± 13.12, 44.35 ± 11.84, 35.06 ± 10.62, and 107.05 ± 14.30, respectively. In the SW579 cell line, the number of invasive cells was 164.33 ± 22.28, 155.67 ± 29.52, 88.23 ± 13.64, 81.06 ± 15.58, and 159.84 ± 20.32, respectively. In the 8505C cell line, the number of invasive cells was 256.76 ± 34.57, 232.06 ± 30.52, 175.74 ± 21.58, 171.06 ± 20.52, and 249.27 ± 27.34, respectively. Amongst the three cell lines, the number of invasive cells was highest in the 8505C cell line, lowest in the K1 cell line, and the SW579 cell line was in between (all *P*<0.05). There was no significant difference in the number of invasive cells in the blank, NC, and LINC00312 overexpression + *miR-197-3p* mimics groups (all *P*>0.05). The number of invasive cells in the LINC00312 overexpression and *miR-197-3p* inhibitors groups were significantly lower than the blank and NC groups. The number of invasive cells in the LINC00312 overexpression group was significantly lower than the LINC00312 overexpression + *miR-197-3p* mimics group (all *P*<0.05). These results reveal that LINC00312 suppresses K1, SW579, and 8505C cell invasion by down-regulating *miR-197-3p*.

**Figure 5:** Invasion abilities of K1, SW579, and 8505C cells amongst five groups (mean ± S.D.) (**A**) cell invasion observed under the optical microscope; (**B**) comparison of the number of invasive cells; *, *P*<0.05, compared with the blank group; ^&^, *P*<0.05 compared with the LINC00312 overexpression + *miR-197-3p* mimics group; four wells of cells in each group were repeated, and the experiment was repeated for three times.

### LINC00312 reduces K1, SW579, and 8505C cell migration by down-regulating *miR-197-3p*

Figure 6 presents the scratch width percentages of each cell line 48 h after transfection in the blank, NC, LINC00312 overexpression, *miR-197-3p* inhibitors, and LINC00312 overexpression + *miR-197-3p* mimics groups (the same below). The K1 cell line percentages were 31.44 ± 2.03, 30.01 ± 3.27, 58.44 ± 7.03, 55.67 ± 6.27, and 27.21 ± 3.83, respectively. The SW579 cell line percentages were 19.41 ± 4.21, 17.43 ± 4.08, 37.32 ± 4.36, 35.77 ± 4.92, and 16.55 ± 1.91, respectively. The 8505C cell line percentages were 10.85 ± 2.34, 8.47 ± 3.57, 23.03 ± 5.01, 21.81 ± 2.57, and 6.03 ± 1.63, respectively. These results demonstrate that the scratch width is narrowest in 8505C cells, widest in K1 cells, and medium in SW579 cells (all *P*<0.05). Scratch width in the LINC00312 overexpression and the *miR-197-3p* inhibitor groups was significantly wider than those of the blank and NC groups. The scratch width in the LINC00312 overexpression group was wider than that of the LINC00312 overexpression + *miR-197-3p* mimics group. These findings indicate that LINC00312 reduces K1, SW579, and 8505C cell migration by down-regulating *miR-197-3p*.

**Figure 6:** Migration abilities of K1, SW579, and 8505C cells amongst five groups (mean ± S.D.) (**A**) Cell migration observed under the optical microscope; (**B**) histogram of cell scratch width in each group; *, *P*<0.05, compared with the blank group; ^#^, *P*<0.05, compared with the NC group; ^&^, *P*<0.05, compared with the LINC00312 overexpression + *miR-197-3p* mimics group; four wells of cells in each group were repeated, and the experiment was repeated for three times.

### LINC00312 inhibits the *in vivo* tumorigenesis of K1, SW579, and 8505C cells by down-regulating *miR-197-3p*

The tumor xenograft results in nude mice are presented in Figure 7. In the LINC00312 overexpression group, tumor size was largest in 8505C cells (689.05 ± 65.61), smallest in K1 cells (239.05 ± 47.91) and SW579 cells were in between (451.82 ± 79.08) (all *P*<0.05). The overexpression of LINC00312 and low expression of *miR-197-3p* significantly weakened the thyroid tumorigenesis of K1, SW579, and 8505C cells in nude mice. There was no significant difference in the tumor size of nude mice in the blank (627.21 ± 113.29), NC (682.21 ± 79.08), and LINC00312 overexpression + *miR-197-3p* mimic groups (649.35 ± 70.54) in the K1, SW579, and 8505C cell lines (all *P*>0.05). In the K1, SW579, and 8505C cells, tumor size in the LINC00312 overexpression (239.05 ± 49.71) and *miR-197-3p* inhibitor groups (221.82 ± 54.37) were significantly smaller than the blank (27.21 ± 113.29) and the NC groups (682.21 ± 79.08) (all *P*<0.05). Tumor size in the LINC00312 overexpression group (239.05 ± 49.71) was significantly smaller than in the LINC00312 overexpression + *miR-197-3p* mimics group (649.35 ± 70.54) (*P*<0.05). The results demonstrate that LINC00312 inhibits the *in vivo* tumorigenesis of K1, SW579, and 8505C cells by down-regulating *miR-197-3p*. The results also reveal that *miR-197-3p* mimics reverse the tumorigenic ability of TC cells.

**Figure 7:** Effects of LINC00312 on thyroid tumorigenesis by down-regulating *miR-197-3p* (mean ± S.D.) (**A**) The tumor measurement of nude mice in each group; (**B**) the tumor size of nude mice in each group; *, *P*<0.05, compared with the blank group; ^#^, *P*<0.05, compared with the NC group; ^&^, *P*<0.05, compared with LINC00312 overexpression + *miR-197-3p* mimics group; four wells of cells in each group were repeated, and the experiment was repeated for three times.

## Discussion

TC is an endocrine malignancy, which usually forms as a result of ionizing radiations [18]. Although death rates associated with TC have declined in most parts of the world, TC incidence has been continuously rising over the recent decades [19]. It has been recently revealed that a relationship exists between TC and lncRNAs such as NR_036575.1 and PVT1. The expression of these lncRNAs contribute to the biological changes in TC cells [5,20]. Our study aims to detect the effect of LINC00312 on TC by regulating *miR-197-3p*. The results demonstrate that LINC00312 overexpression can inhibit the proliferation, migration and invasion of TC cells by down-regulating the expression of *miR-197-3p*.

Most importantly, the present study indicated that TC tissues have a lower expression of LINC00312 and a higher expression of *miR-197-3p* than the adjacent normal tissues. The role of miRNAs and lncRNAs during the transcription and post-transcriptional stages has been widely acknowledged [21]. LncRNAs aberrant expression in human cancer tissues may be correlated with tumor metastasis and disease prognosis [22]. In addition, Yang et al. [23] revealed that the altered expression of lncRNAs can induce gene aberrant expression and tumorigenesis in human papillary TC. Zhang et al. [10] advocated that there is a low LINC00312 expression in nasopharyngeal carcinoma. A recent study conducted by Wang et al. elucidated that LINC00312 is negatively associated with *miR-197-3p* in bladder cancer [14]. Our study also found a relatively high expression of LINC00312 and low expression of *miR-197-3p* in normal tissues [14]. In TC specimens, the up-regulation of *miR-197-3p* may be regulated by LINC00312 through its endogenous RNA or miRNA sponges [22].

In addition, the present study highlights that a low expression of LINC00312 may appear in patients with lymphatic metastasis, in TNM stage III/IV or have larger tumor diameters. Conversely, *miR-197-3p* is expressed highly in patients with such clinicopathological characteristics. In nasopharyngeal carcinoma, LINC00312 was revealed to be positively correlated with lymphatic metastasis and negatively correlated with tumor diameter [10]. Moreover, according to Sun et al. [20], lncRNA NR_036575.1 is significantly correlated with tumor diameter and extrathyroidal extension in papillary TC. Furthermore, the results indicate that the expression levels of LINC00312 and *miR-197-3p* are related to TC tissue-type. Therefore, LINC00312 and *miR-197-3p* may be assistant proofs for detecting TC clinicopathological characteristics.

Moreover, it was demonstrated that LINC00312 overexpression can weaken the migration, invasion, and tumorigenesis ability (*in vivo*) of TC cells by down-regulating *miR-197-3p*. Additionally, the expression level of p120 was proved to be negatively correlated with *miR-197-3p* expression and positively correlated with LINC00312 expression. This further validates the role of LINC00312 and *miR-197-3p* in TC cells. We confirmed that p120 is a direct target gene of *miR-197-3p. MiR-197-3p* is a mature body of *miR-197*, and *miR-197* is associated with the expression of various tumor-suppressor genes such as *FUS1* and *NLK* [24,25]. Hamada et al. [26] stated that *miR-197* directly targets p120 through the transient expression of *miR-197* and the 3′-UTR assay of p120 mRNA. Additionally, a lack of p120 is likely to increase the risk of cancer cell migration and invasion in the buccal cavity, gullet, and fore stomach. This is due to the fact that p120 mediates cadherin constancy and turnover [27]. Moreover, *miR-197-3p* overexpression in ovarian cancer can stimulate cancer cell (A2780) proliferation and invasion [25]. MiR-197-3p has also been shown to facilitate pancreatic cancer cells invasion and migration [26]. A recent study indicated that LINC00312 can suppress the invasion and metastasis of bladder cancer cell by directly mediating *miR-197-3p* [14]. Therefore, we hypothesize that LINC00312 can inhibit the migration, invasion, and tumorigenesis abilities of TC cells indirectly by regulating p120 and *miR-197-3p*.

According to the transwell and scratch test, the 8505C cell line (anaplastic TC) had the strongest invasion and migration abilities, K1 (papillary TC) had the weakest, and SW579 (squamous TC) was in between. Anaplastic TC is a highly aggressive malignancy [28], whereas K1 papillary TC is well differentiated and has a good prognosis [29]. Squamous TC is an aggressive neoplasm which has a bad prognosis [30]. In terms of differentiation, 8505C is undifferentiated, K1 is well differentiated, and SW579 is poorly differentiated. The results observed may be caused by the negative correlation between the invasion and migration ability, and the degree of cell differentiation.

Overall, we demonstrated that the migration and invasion of TC cells can be suppressed by LINC00312 overexpression by down-regulating *miR-197-3p*. Our study also indicated that LINC00312 and *miR-197-3p* may be potential therapeutic targets for TC. However, TC is influenced by various genes through a complex mechanism. Additionally, the sample size of research which studied the clinicopathological features of TC was limited. Therefore, the exact monocular mechanism behind LINC00312 effect on *miR-197-3p* is still awaiting further specific research.

## Abbreviations

DMEM: Dulbecco’s modified Eagle’s medium
LARII: luciferase assay reagent II
LINC00312: long intergenic noncoding RNA LINC00312
lncRNA: long noncoding RNA
LSD-t: least significant differenc
NC: negative control
OD: optical density
qRT-PCR: quantitative real-time PCR
TBST: Tribs-buffered saline Tween-20
TC: thyroid cancer
TNM: tumor node metastasis
WT: wild-type
